The article "MMP-3 and MMP-8 single-nucleotide polymorphisms are related to alcohol-induced osteonecrosis of the femoral head in Chinese males" was published in 2017. Journal: Oncotarget.

# *MMP-3* and *MMP-8* single-nucleotide polymorphisms are related to alcohol-induced osteonecrosis of the femoral head in Chinese males

**DOI:** 10.18632/oncotarget.15587

**Published:** 2017-02-21

**Authors:** Junyu Chen, Wanlin Liu, Yuju Cao, Xiyang Zhang, Yongchang Guo, Yong Zhu, Jian Li, Jieli Du, Tianbo Jin, Guoqiang Wang, Jianzhong Wang

**Affiliations:** ^1^ Inner Mongolia Medical University, Hohhot, Inner Mongolia 010030, China; ^2^ Department of the 2nd Affiliated Hospital of Inner Mongolia Medical University, Hohhot, Inner Mongolia 010030, China; ^3^ Zhengzhou Traditional Chinese Medicine Traumatology Hospital, Zhengzhou, Henan 450016, China; ^4^ School of Life Sciences, Northwest University, Xi’an, Shaanxi 710069, China; ^5^ Key Laboratory of Molecular Mechanism and Intervention Research for Plateau Diseases of Tibet Autonomous Region, School of Medicine, Xizang Minzu University, Xianyang, Shaanxi 712082, China; ^6^ Key Laboratory of High Altitude Environment and Genes Related to Diseases of Tibet Autonomous Region, School of Medicine, Xizang Minzu University, Xianyang, Shaanxi 712082, China; ^7^ Key Laboratory for Basic Life Science Research of Tibet Autonomous Region, School of Medicine, Xizang Minzu University, Xianyang, Shaanxi 712082, China

**Keywords:** *MMP-3*, *MMP-8*, alcohol-induced osteonecrosis of the femoral head, genetic, single-nucleotide polymorphism

## Abstract

Our study investigated the association between *MMP-3* and *MMP-8* single-nucleotide polymorphisms (SNPs) and alcohol-induced osteonecrosis of the femoral head (ONFH) in 695 Chinese males (299 cases and 396 control subjects). The minor allele of *MMP-3* rs650108 was associated with a 0.78-fold decrease in alcohol-induced ONFH risk in the allelic model (95% CI = 0.63-0.97, *P* = 0.026). In the genetic model adjusted for age, rs650108 was associated with decreased risk of alcohol-induced ONFH in the dominant model (OR = 0.68, 95% CI = 0.49-0.95, *P* = 0.022) and log-additive model (OR = 0.78, 95% CI = 0.63-0.98, *P* = 0.030); *MMP-8* rs11225394 was associated with increased risk in the codominant model (OR = 1.72, 95% CI = 1.15-2.58, *P*= 0.010), dominant model (OR = 1.67, 95% CI = 1.12-2.48, *P* = 0.012), over-dominant model (OR = 1.73, 95% CI = 1.16-2.59, *P* = 0.007) and log-additive model (OR = 1.57, 95% CI= 1.07-2.32, *P* = 0.022); and *MMP-8* rs2012390 was associated with decreased risk in the dominant model (OR = 0.72, 95% CI = 0.53-0.97, *P* = 0.032) and log-additive model (OR = 0.77, 95% CI = 0.60-0.98, *P* = 0.035). Haplotype analysis showed that the CGATATGT sequence mediated decreased alcohol-induced ONFH risk (OR = 0.75, 95% CI = 0.57-0.97, *P* = 0.029). Therefore, among Chinese males, *MMP-3* rs650108 and *MMP-8* rs2012390 decrease alcohol-induced ONFH risk and *MMP-8* rs11225394 increases it. Further study is needed to validate our conclusion.

## INTRODUCTION

Alcohol-induced osteonecrosis of the femoral head (ONFH) is a degenerative lesion of joints and a partial blood circulation disorder of the femoral head. It has several complex causes that are common to non-traumatic ONFH and results in further osteocyte ischemia, necrosis, bone trabecula fracture, and complete collapse of the femoral head [1]. It causes a destructive femoral head collapse in approximately 80% of patients without treatment [2, 3]. Because drinking has become a global health concern, the World Health Organization (WHO) has identified high alcohol consumption as one of the most important pathogenic factors of alcohol-induced ONFH (http://www.who.int/entity/substanceabuse/publications/globalalcoholreport/msbgsrwpr.pdf), and the incidence of this disease is rising worldwide. For example, the overall number of osteonecrosis cases in China has almost reached 7 million and 100,000 to 200,000 new patients are diagnosed each year [4], approximately one-third of whom have alcohol-induced ONFH. This multifactorial disease is the result of several complicated interactions among environmental, lifestyle, metabolic and genetic factors [5–7]. The widely known pathologic mechanisms of alcohol-induced ONFH are dyslipidemia, osteoporosis, intraosseous hypertension, gene-associated mechanisms, and the abnormal differentiation of osteoblasts/osteoclasts from bone marrow mesenchymal stem cells (BMSCs), and most of the mechanisms are related to the pathologic process of dyslipidemia. So, more investigation of the pathologic mechanisms of alcohol-induced ONFH from different perspectives is needed. Genetic research offers insight into the occurrence, treatment and development of alcohol-induced ONFH, and genetic variations are identified as a normal biological phenomenon that influences immunoreaction and protein transcription and even determine individual susceptibilities of some pathological diseases of the joints [8–10]. Although many people drink, only some of them experience alcohol-induced ONFH, illustrating that individual susceptibilities might cause different incidences of this disease among different populations. Single-nucleotide polymorphisms (SNPs) have been widely researched because of their variations in a single base pair in the DNA sequence. On the basis of previous studies, we found the polymorphisms of several genes, including *ApoA1*, *ApoB*, *SREBF1* and *TLR4* were associated with the risk of alcohol-induced ONFH [4, 11–13].

Matrix metalloproteinases (MMPs) are a family of proteases that could be involved in the degradation of osseous tissue and other extracellular matrices in the human body. Among the more than 20 types of MMP genes, *MMP-3* and *MMP-8* are the most influential. *MMP-3* encodes an enzyme that degrades fibronectin, laminin, collagens III, IV, IX, and X, and cartilage proteoglycans [14]. *MMP-8* is involved in the breakdown of the extracellular matrix in embryonic development, reproduction, and tissue remodeling [15]. Previous studies show that several types of *MMPs* are abnormally expressed in different orthopedic diseases. *MMP-1* and *MMP-3* are overexpressed in the synoviocytes and chondrocytes of osteoarthritis patients. *MMP-2* and *MMP-9* are overexpressed in the serum and synovia of osteoarthritis patients [16]. Collectively, the dynamic equilibrium of MMPs and their natural inhibitors, tissue inhibitors of metalloproteinases (TIMPs), can significantly influence bone metabolism in the human body [17]. However, no studies have explored the relation between *MMP-3* and *MMP-8* in the MMP/TIMP pathway and alcohol-induced ONFH. Our case-control study investigated whether *MMP-3* and *MMP-8* have a potential association with alcohol-induced ONFH among a population of Chinese males at a genetic level.

## RESULTS

We performed a case-control study that selected 695 individuals, including 299 alcohol-induced ONFH patients (mean age: 43.24 ± 13.07) and 396 healthy control subjects (mean age: 47.62 ± 10.28). All the individuals are males (Table 1). We researched eight SNPs (rs639752, rs650108, rs520540, rs646910, rs602128, rs679620, rs678815, and rs522616) on gene *MMP-3* and five SNPs (rs3740938, rs2012390, rs1940475, rs11225394, and rs11225395) on gene *MMP-8*. The basic SNP information of all the individuals in our study, including the minor allele frequency (MAF), odds ratios (ORs), 95% confidence intervals (95% CIs), position, band, alleles, and the *P-*values of alleles evaluated by χ^2^ test, are shown in Table 2. All 13 SNPs are in accord with the Hardy-Weinberg equilibrium (HWE) (*P* > 0.05). The minor allele G of rs650108 on *MMP-3* was significantly associated with 0.78-fold decreased alcohol-induced ONFH risk (OR = 0.78, 95% CI = 0.63-0.97, *P* = 0.026). All the primers utilized for genotyping in this study are listed in Table 7, and the statistical power of the SNPs in our study are listed in the Table 8.

**Table 1:** Characteristics of the male individuals in controls and alcohol-induced ONFH

	Group	N	Mean	Std. Deviation	Mean±SD	*P*-value
Age	Case	299	43.24	13.07	43.24±13.07	*P* < 0.001*
	Control	396	47.62	10.28	47.62±10.28	

* *P* values was calculated by Welch's t-tests

**Table 2:** Basic SNP information summary of all the male individuals in our study

Gene	SNP ID	Position	Band	Alleles A^a^/B	MAF		Role	HWE-*P*	OR(95%CI)	*P*^b^ value
					Case	Control				
MMP-3	rs639752	102707339	11q22.3	C/A	0.31	0.36	Intron	0.27	0.82(0.65-1.02)	0.079
MMP-3	rs650108	102708787	11q22.3	G/A	0.39	0.45	Intron	0.54	0.78(0.63-0.97)	0.026*
MMP-3	rs520540	102709425	11q22.3	A/G	0.31	0.36	Coding exon	0.27	0.82(0.65-1.02)	0.079
MMP-3	rs646910	102709522	11q22.3	A/T	0.08	0.09	Intron (boundary)	0.76	0.83(0.57-1.23)	0.354
MMP-3	rs602128	102713465	11q22.3	A/G	0.31	0.36	Coding exon	0.51	0.83(0.66-1.04)	0.104
MMP-3	rs679620	102713620	11q22.3	T/C	0.31	0.36	Coding exon	0.44	0.81(0.65-1.02)	0.074
MMP-3	rs678815	102713777	11q22.3	G/C	0.31	0.36	Intron	0.33	0.81(0.65-1.02)	0.075
MMP-3	rs522616	102715048	11q22.3	C/T	0.39	0.34	Promoter	1.00	1.24(1.00-1.55)	0.054
MMP-8	rs3740938	102587062	11q22.3	A/G	0.23	0.26	Coding exon	0.70	0.83(0.64-1.06)	0.134
MMP-8	rs2012390	102590777	11q22.3	G/A	0.26	0.3	Intron	0.48	0.79(0.63-1.01)	0.058
MMP-8	rs1940475	102593248	11q22.3	T/C	0.36	0.39	Coding exon	1.00	0.90(0.73-1.13)	0.371
MMP-8	rs11225394	102595413	11q22.3	T/C	0.11	0.08	Intron (boundary)	1.00	1.42(0.98-2.05)	0.059
MMP-8	rs11225395	102596480	11q22.3	A/G	0.35	0.38	Promoter	1.00	0.90(0.72-1.12)	0.336

SNP, single nucleotide polymorphism; MAF, minor allele frequency; HWE, Hardy-Weinberg equilibrium; ORs, odds ratios; CI, confidence interval;

^a^ Minor allele

^b^ *P* were adjusted by gender and age, * *P* < 0.05, statistical significance

We developed a hypothesis that compared each minor allele with the corresponding wild-type allele. Every minor allele on an SNP was one risk factor, and we built five different genetic models and used unconditional logistic regression to assess the relation between SNPs and alcohol-induced ONFH risk. The results are shown in Table 3 . We found that rs650108 on *MMP-3* was related to a decreased risk of alcohol-induced ONFH in the dominant model (OR = 0.69, 95% CI = 0.50-0.95, *P* = 0.023) and the log-additive model (OR = 0.78, 95% CI = 0.63-0.97, *P* = 0.025). We also found that rs11225394 on *MMP-8* was related to an increased alcohol-induced ONFH risk in the codominant model (OR = 1.59, 95% CI = 1.08-2.36, *P* = 0.021), the dominant model (OR = 1.54, 95% CI = 1.04-2.27, *P* = 0.030), and the over-dominant model (OR = 1.60, 95% C I = 1.08-2.38, *P* = 0.018).

**Table 3:** Analysis of the association between SNPs and alcohol-induced ONFH risk in males (based on logistical tests)

SNP ID	Model	Genotype	Group=control	Group=Alcohol	OR (95% CI)	*P*-value	AIC	BIC
rs650108 (MMP-3)	Codominant	A/A	116 (29.4%)	112 (37.6%)	1	0.064	947.6	961.2
		A/G	202 (51.1%)	139 (46.6%)	0.71 (0.51-1.00)			
		G/G	77 (19.5%)	47 (15.8%)	0.63 (0.40-0.99)			
	Dominant	A/A	116 (29.4%)	112 (37.6%)	1	0.023*	945.9	955
		A/G-G/G	279 (70.6%)	186 (62.4%)	0.69 (0.50-0.95)			
	Recessive	A/A-A/G	318 (80.5%)	251 (84.2%)	1	0.200	949.5	958.5
		G/G	77 (19.5%)	47 (15.8%)	0.77 (0.52-1.15)			
	Overdominant	A/A-G/G	193 (48.9%)	159 (53.4%)	1	0.240	949.7	958.8
		A/G	202 (51.1%)	139 (46.6%)	0.84 (0.62-1.13)			
	Log-additive	---	---	---	0.78 (0.63-0.97)	0.025*	946.1	955.2
rs11225394 (MMP-8)	Codominant	C/C	327 (84.7%)	234 (78.3%)	1	0.021*	936.8	950.4
		T/C	57 (14.8%)	65 (21.7%)	1.59 (1.08-2.36)			
		T/T	2 (0.5%)	0 (0%)	0.00 (0.00-NA)			
	Dominant	C/C	327 (84.7%)	234 (78.3%)	1	0.030*	937.8	946.9
		T/C-T/T	59 (15.3%)	65 (21.7%)	1.54 (1.04-2.27)			
	Recessive	C/C-T/C	384 (99.5%)	299 (100%)	1	0.130	940.2	949.3
		T/T	2 (0.5%)	0 (0%)	0.00 (0.00-NA)			
	Overdominant	C/C-T/T	329 (85.2%)	234 (78.3%)	1	0.018*	937	946
		T/C	57 (14.8%)	65 (21.7%)	1.60 (1.08-2.38)			
	Log-additive	---	---	---	1.46 (1.00-2.13)	0.052	938.8	947.8

SNP, single nucleotide polymorphism; ORs, odds ratios; CI, confidence interval; AIC, Akaike's Information criterion; BIC, Bayesian Information criterion.

*P* value was calculated with logistic analysis. * *P* < 0.05, statistical significance.

Furthermore, we found that the results were still superior after adjusting for age, and we also found another SNP (rs2012390) on *MMP-8* that was significant but not superior. After adjusting for age, we found, as shown in Table 4, that rs650108 on *MMP-3* was associated with a decreased alcohol-induced ONFH risk in the dominant model (OR = 0.68, 95% CI = 0.49-0.95, *P* = 0.022) and the log-additive model (OR = 0.78, 95% CI = 0.63-0.98, *P* = 0.030), and rs11225394 on *MMP-8* was associated with an increased risk of alcohol-induced ONFH in the codominant model (OR = 1.72, 95% CI = 1.15-2.58, *P* = 0.010), the dominant model (OR = 1.67, 95% CI = 1.12-2.48, *P* = 0.012), the over-dominant model (OR = 1.73, 95% CI = 1.16-2.59, *P* = 0.007), and the log-additive model (OR = 1.57, 95% CI = 1.07-2.32, *P* = 0.022). Additionally, we found that rs2012390 on *MMP-8* was significant and associated with a decreased alcohol-induced ONFH risk in the dominant model (OR=0.72, 95% CI = 0.53-0.97, *P* = 0.032) and the log-additive model (OR = 0.77, 95% CI = 0.60-0.98, *P* = 0.035).

**Table 4:** Analysis of the association between SNPs and alcohol-induced ONFH risk in males (adjusted for age)

SNP ID	Model	Genotype	Group=control	Group=Alcohol	OR (95% CI)	*P*-value	AIC	BIC
rs650108 (MMP-3)	Codominant	A/A	116 (29.4%)	112 (37.6%)	1	0.066	925.6	943.7
		A/G	202 (51.1%)	139 (46.6%)	0.70 (0.49-0.98)			
		G/G	77 (19.5%)	47 (15.8%)	0.64 (0.41-1.01)			
	Dominant	A/A	116 (29.4%)	112 (37.6%)	1	0.022*	923.7	937.3
		A/G-G/G	279 (70.6%)	186 (62.4%)	0.68 (0.49-0.95)			
	Recessive	A/A-A/G	318 (80.5%)	251 (84.2%)	1	0.270	927.8	941.4
		G/G	77 (19.5%)	47 (15.8%)	0.80 (0.53-1.19)			
	Overdominant	A/A-G/G	193 (48.9%)	159 (53.4%)	1	0.190	927.2	940.9
		A/G	202 (51.1%)	139 (46.6%)	0.81 (0.60-1.11)			
	Log-additive	---	---	---	0.78 (0.63-0.98)	0.030*	924.3	937.9
rs2012390 (MMP-8)	Codominant	A/A	189 (47.7%)	165 (55.4%)	1	0.095	928.2	946.4
		A/G	174 (43.9%)	113 (37.9%)	0.73 (0.53-1.00)			
		G/G	33 (8.3%)	20 (6.7%)	0.65 (0.36-1.19)			
	Dominant	A/A	189 (47.7%)	165 (55.4%)	1	0.032*	926.4	940
		A/G-G/G	207 (52.3%)	133 (44.6%)	0.72 (0.53-0.97)			
	Recessive	A/A-A/G	363 (91.7%)	278 (93.3%)	1	0.330	930	943.6
		G/G	33 (8.3%)	20 (6.7%)	0.75 (0.42-1.35)			
	Overdominant	A/A-G/G	222 (56.1%)	185 (62.1%)	1	0.100	928.2	941.9
		A/G	174 (43.9%)	113 (37.9%)	0.77 (0.56-1.05)			
	Log-additive	---	---	---	0.77 (0.60-0.98)	0.035*	926.5	940.1
rs11225394 (MMP-8)	Codominant	C/C	327 (84.7%)	234 (78.3%)	1	0.001*	914.9	933
		T/C	57 (14.8%)	65 (21.7%)	1.72 (1.15-2.58)			
		T/T	2 (0.5%)	0 (0%)	0.00 (0.00-NA)			
	Dominant	C/C	327 (84.7%)	234 (78.3%)	1	0.012*	915.8	929.4
		T/C-T/T	59 (15.3%)	65 (21.7%)	1.67 (1.12-2.48)			
	Recessive	C/C-T/C	384 (99.5%)	299 (100%)	1	0.140	920	933.5
		T/T	2 (0.5%)	0 (0%)	0.00 (0.00-NA)			
	Overdominant	C/C-T/T	329 (85.2%)	234 (78.3%)	1	0.007*	914.8	928.4
		T/C	57 (14.8%)	65 (21.7%)	1.73 (1.16-2.59)			
	Log-additive	---	---	---	1.57 (1.07-2.32)	0.022*	916.9	930.5

ORs, odds ratios; CI, confidence interval; AIC, Akaike's Information criterion; BIC, Bayesian Information criterion.

*P* value was adjusted by age and gender; * *P* < 0.05, statistical significance.

Our study used polymorphism detection to analyze the pairwise linkage disequilibrium (LD) of *MMP-3* and *MMP-8*. The parameters r^2^ and D′ were used to analyze the LD pattern, and the results are shown in Figure 1 and Table 5 . We observed one block in *MMP-3*, including eight SNPs: rs639752, rs650108, rs520540, rs646910, rs602128, rs679620, rs678815, and rs522616. We used χ^2^ and logistic tests to analyze the haplotype (Table 5). The CGATATGT sequence was found to be associated with a significantly decreased alcohol-induced ONFH risk after adjustment for age (OR = 0.75, 95% CI = 0.57-0.97, *P* = 0.029). Additionally, we did not find any association between alcohol-induced ONFH and *MMP-8* after analyzing the pairwise LD, the results are shown in Table 6 and Figure 2.

**Figure 1:** We used the parameters r2 and D′ to analyze the linkage disequilibrium (LD) of the SNPs on *MMP-3* Significant LD is indicated by bright red standard colors.

**Table 5:** Haplotype association with response (n=695, adjusted by age)

	rs639752	rs650108	rs520540	rs646910	rs602128	rs679620	rs678815	rs522616	Freq	OR (95% CI)	*P*-value
1	A	A	G	T	G	C	C	C	0.3655	1	---
2	C	G	A	T	A	T	G	T	0.3367	0.75 (0.57 - 0.97)	0.029*
3	A	A	G	T	G	C	C	T	0.2079	0.88 (0.65 - 1.18)	0.380
4	A	G	G	A	G	C	C	T	0.0849	0.75 (0.50 - 1.14)	0.190
rare	*	*	*	*	*	*	*	*	0.005	0.47 (0.08 - 2.75)	0.400

Global haplotype association *P*-value: 0.19

rs639752, rs650108, rs520540, rs646910, rs602128, rs679620, rs678815 and rs522616 are on gene *MMP-3*

ORs, odds ratios; CI, confidence interval;

* *P* < 0.05, statistical significance.

**Table 6:** Haplotype association with response (n=695, adjusted by age)

	rs3740938	rs2012390	rs1940475	rs11225394	rs11225395	Freq	OR (95% CI)	*P*-value
1	G	A	C	C	G	0.6226	1	---
2	A	G	T	C	A	0.2457	0.81 (0.62 - 1.05)	0.12
3	G	A	T	T	A	0.0928	1.37 (0.93 - 2.03)	0.11
4	G	G	T	C	A	0.0267	0.55 (0.26 - 1.13)	0.11
5	G	G	T	C	G	0.0108	1.02 (0.35 - 2.97)	0.97

Global haplotype association *p*-value: 0.021

**Table 7:** All the information of the primers in this case-control study

Gene	SNP _ID	1st-PCR primer sequences	2nd-PCR primer sequences	UEP sequences
MMP-3	rs639752	ACGTTGGATGCAGATAAATTCTCCACTTGC	ACGTTGGATGGGCTGCAATGCAGGGAAAAG	tGGGAAGAAAGAAATAGGTGAT
MMP-3	rs650108	ACGTTGGATGGTCACTGTCTCATTGTGTGT	ACGTTGGATGTCAGGTAGAGGTGACAAGTG	tAAGTGGGTGAGGTTAGA
MMP-3	rs520540	ACGTTGGATGGCGAAAGGGCTTAACTGTTAT	ACGTTGGATGCCAGCTCGTACCTCATTTCC	CTCGTACCTCATTTCCTCTGAT
MMP-3	rs646910	ACGTTGGATGCCACTGTAAGCTGGTGACTA	ACGTTGGATGGTTAAGCCCTTTCGCTTTAG	CGCTTTAGAAATACACTTTAGCATCT
MMP-3	rs602128	ACGTTGGATGCTTCGGGATGCCAGGAAA	ACGTTGGATGAAGCTGGACTCCGACACTCT	CAGGTGTGGAGTTCCTGA
MMP-3	rs679620	ACGTTGGATGAACAGGACCACTGTCCTTTC	ACGTTGGATGAGAAATATCTAGAAAACTAC	tcTCTAGAAAACTACTACGACCTC
MMP-3	rs678815	ACGTTGGATGAATGCAACGTAATTTTAGC	ACGTTGGATGTGGAGTATTTCTCTAGCTTG	TCTCTAGCTTGCTGAAATAATG
MMP-3	rs522616	ACGTTGGATGCGTAGCTGCTCCATAAATAG	ACGTTGGATGACAGAGAGAATTTCAGTCCG	gaCGGTAAGCAATGTAATTCATTTCA
MMP-8	rs3740938	ACGTTGGATGGTCAGTAAGAGGAATCAAAG	ACGTTGGATGTGACATTTGATGCTATCAC	GATGCTATCACCACACT
MMP-8	rs2012390	ACGTTGGATGACTGTTTCTAGGTCACACCC	ACGTTGGATGTCAGGGAGAGGAAGCAATTC	gAAGCAAATGTGAGGAAGAT
MMP-8	rs1940475	ACGTTGGATGTTTGGGTTGAATGTGACGGG	ACGTTGGATGTAAAACCACCACTGTCAGGC	CTCCACAGCGAGGCTTTT
MMP-8	rs11225394	ACGTTGGATGCAATCTCAAACTAATCACCC	ACGTTGGATGTTAGGAAATAGTGTGGGTTG	AGTGTGGGTTGTTTTCTCTT
MMP-8	rs11225395	ACGTTGGATGAGAGCTGCTGCTCCACTATG	ACGTTGGATGGTTTAGAGAGACTGAGCTGG	gCTGAGCTGGGAGCTACTATA

**Table 8:** All the statistical power of the SNPs in this study

SNP_ID	Gene(s)	case _n1	control _n2	case _A	control _A	case _p1	contol _p2	p	zβ	power
rs639752	MMP3	598	792	186	186	0.311037	0.234848	0.267626	1.206173	**0.886124538**
rs650108	MMP3	596	790	233	233	0.39094	0.294937	0.336219	1.777753	**0.962277821**
rs520540	MMP3	598	792	186	186	0.311037	0.234848	0.267626	1.206173	**0.886124538**
rs646910	MMP3	598	792	46	46	0.076923	0.058081	0.066187	-0.55131	0.290709864
rs602128	MMP3	596	782	187	187	0.313758	0.23913	0.271408	1.117555	**0.868121497**
rs679620	MMP3	598	792	187	187	0.312709	0.236111	0.269065	1.217832	**0.88835615**
rs678815	MMP3	592	790	185	185	0.3125	0.234177	0.267728	1.282388	**0.900146697**
rs522616	MMP3	598	790	236	236	0.394649	0.298734	0.340058	1.768172	**0.961483907**
rs3740938	MMP8	598	790	135	135	0.225753	0.170886	0.194524	0.590001	0.722404948
rs2012390	MMP8	596	792	153	153	0.256711	0.193182	0.220461	0.85629	**0.804081313**
rs1940475	MMP8	598	792	217	217	0.362876	0.27399	0.31223	1.571273	**0.941940363**
rs11225394	MMP8	598	772	65	65	0.108696	0.084197	0.094891	-0.41971	0.337347429
rs11225395	MMP8	598	792	210	210	0.351171	0.265152	0.302158	1.488018	**0.931626918**

**Figure 2:** We used the parameters r2 and D′’ to analyze the linkage disequilibrium (LD) of the SNPs on *MMP-8* Significant LD is indicated by bright red standard colors.

## DISCUSSION

Excessive and chronic alcohol consumption are the most important causes of alcohol-induced ONFH. The association between several polymorphisms and alcohol-induced ONFH has been reported [4, 11, 13, 18]]. However, each polymorphism only contributes to a small relative risk of alcohol-induced ONFH, and more comprehensive genetic polymorphisms are needed to enrich the genetic information on this disease. Our study is the first to investigate the association between the *MMP-3* and *MMP-8* polymorphisms and alcohol-induced ONFH. We researched 13 SNPs on *MMP-3* and *MMP-8*, and found two protective SNPs, rs650108 (10556C>T) on *MMP-3* and rs2012390 (9909C>T), on *MMP-8* and one high-risk SNP, rs11225394 (5273G>A), on *MMP-8* associated with alcohol-induced ONFH risk.

The destruction and repair of bone tissue depend on bone resorption and bone formation. They are the basis of bone metabolism. MMPs are a group of endopeptidases that contain zinc finger motifs, which have the function of degrading all the components of extracellular matrix. A study by Grässel et al [19] reported that the expression and activity of *MMP-2* and *MMP-9* increase the impaired bone matrix repair capacity, restoring the balance between bone resorption and de novo bone formation in ONFH. So *MMP-3* and *MMP-8*, might be like *MMP-2* and *MMP-9* and are associated with ONFH.

*MMP-3* and *MMP-8* localize to chromosome 11q22.3. *MMP-3* encodes an enzyme that degrades fibronectin, laminin, collagens III, IV, IX, and X, and cartilage proteoglycans. The expression of *MMP-3* involves in the degradation of bone matrix in bone resorption [14]. A previous study demonstrated that 6A/6A polymorphism of *MMP-3* is associated with the degradation of collagen, resulting in extracellular matrix degradation, ultimately leading to cartilage and bone loss [20], and this pathway is one of the major pathological mechanismsmechanism in ONFH. Our research found that rs650108 (10556C>T) of *MMP-3* decreases the risk of alcohol-induced ONFH. We speculated that the polymorphism of *MMP-3* might be involvedinvolve in the prevention pathway of extracellular matrix degradation and decreasing cartilage and bone loss in ONFH. *MMP-8* encodes interstitial collagenases that promote bone tissue degradation. The expression of *MMP-8* involves in the breakdown of extracellular matrix in bony tissue development, reproduction, and tissue remodeling, including disease processes such as arthritis and metastasis [15]. Our research found that rs2012390 (9909C>T) on *MMP-8* decreases ONFH risk and rs11225394 (5273G>A) on *MMP-8* increases ONFH risk. The polymorphisms of *MMP-8* might influence the breakdown pathway of the extracellular matrix in bony tissue development, reproduction, and tissue remodeling, and is a risk or preventionprevent factor in ONFH. Previous studies have determined that *MMP-3* and *MMP-8* are key factors in the pathological process of orthopedic diseases [16, 21, 22]. For example, *MMP-1* and *MMP-3* encode the key enzyme for bone surface collagen formation. The expression of *MMP-1* and *MMP-3* promote bone resorption to accelerate sclerotin repair [23]. In osteoarthritis patients, *MMP-3* promotes the degradation of bone matrix and stimulates bone tissue repair [16]. We speculated that the SNPs rs650108 (10556C>T) on *MMP-3* and rs2012390 (9909C>T) on *MMP-8* might decrease alcohol-induced ONFH risk by regulating the breakdown of the extracellular matrix (ECM) and finally result in regulating bone tissue repair.; We also found rs11225394 (5273G>A) on *MMP-8*increases alcohol-induced ONFH risk. Thethe role of *MMP-3* is supposedly related to the breakdown of the ECM, resulting in the loss of tissue integrity [24].Additionally, *MMP-3* is a factor in the formation of bone tissue and in the formation of osteoclasts, osteoblasts, osteoid and pro-osteoclasts [25]. Osteoclasts are differentiated from pro-osteoclasts, and the dynamic equilibrium of the osteoblast/osteoclast ratio is the major part of the maintenance of bone resorption, bony remodeling, and bone metabolism. We found that the genetic polymorphisms of *MMP-3*, rs650108 (10556C>T), decrease ONFH risk.We speculated that thethe polymorphism of *MMP-3* might on the one hand regulate the breakdown of the ECM and on the other hand influence the formation of osteoblasts and osteoclasts and influence bone metabolism, resulting in decreased alcohol-induced ONFH risk. *MMP-8* is mainly produced by neutrophils and is also expressed by extensive cells, including chondrocytes [26] and synovial fibroblasts [27]. *MMP-8* is a key factor in the pathogenesis of several inflammatory conditions because is encodes a potent collagenolytic enzyme [28]. The action of *MMP-8* in the inflammatory process depends on the stimulus in different situations, and *MMP-8* might have a promoting or protective function in arthritis pathogenesis [29, 30]. A previous investigation indicated that the polymorphism of *MMP-8* influencesinfluence the development of the inflammatory reaction itself [31]. A lack of *MMP-8* causes the aggravation of arthritis through promotion of inflammation by IL-1β and PTX3, inducing the maturation and activation of osteoclasts or enhancement of the inflammatory infiltrate by PROKR2 and IL-1β [32]. So, we speculated that the polymorphisms of *MMP-8* mightmight influence the development of the inflammatory reaction process in the femoral head, and might be involvedand involve in the regulation of the inflammatory response in the bone joint tissue, resulting in an influence on the risk of alcohol-induced ONFH. Additionally, rs650108 (10556C>T) is a sensitive SNP in *MMP-3* that has been found to have an association with the risk of primary sclerosing cholangitis [33], breast cancer [34], and rotator cuff repair [35]. The mutation of rs650108 in these diseases are a key factor in inflammatory or fibrogenic response, and the pathogenic development of alcohol-induced ONFH is closely tied to the fibrogenic response of bone resorption and remodeling of bone tissue. Thus, we speculated that the mutation of rs650108 on *MMP-3* may influence the process of bone resorption and remodeling that is associated with the fibrogenic response in alcohol-induced ONFH. MoreoverMoreover, we found the expression of a different genotype in a different SNP on the same gene might have a different influence in the same disease.

Furthermore, our study is the first to explore the association between alcohol-induced ONFH and *MMP-3* and *MMP-8* polymorphism. Further explorations with larger samples and individuals from different areas are needed to confirm our conclusion.

## MATERIALS AND METHODS

### Ethics committee statement

Our present study strictly observed the principles of the Declaration on Helsinki of the World Medical Association and was approved by the Ethics Committee of Zhengzhou Traditional Chinese Medicine Traumatology Hospital. Informed consent forms were signed by all the individuals and they were all notified for our case-control study.

### Research subjects

Our case-control study consecutively recruited a total of 695 male individuals (299 alcohol-induced ONFH patients and 396 healthy control subjects) from September 2014 to January 2016 in Zhengzhou Traditional Chinese Medicine Traumatology Hospital. All the participants were selected randomly without age restriction and were genetically unrelated ethnic Han Chinese males.

Medical diagnostic criteria of alcohol-induced ONFH is based on clinical manifestations such as pain and activity limitation of hip and sick-side lower limb muscle atrophy. Further diagnosis depends on magnetic resonance imaging (MRI) analysis and examination of changes on X-ray, such as high density shadows of the femoral head, hip joint narrowness and bumpiness, or joint surface rupture. All the selected patients were given thorough physical examinations.

When we selected the participants for the case group, the exclusion criteria were refusal to participate in this study, liver disease or dyslipidemia caused by drugs, not satisfying alcohol-induced ONFH medical diagnostic criteria or the presence of traumatic osteonecrosis or other hip diseases, requirement of steroids for replacement therapy in serious primary disease, and overuse of steroids or a chronic metabolic disorder of the heart, kidney, or liver.

When we selected the control group, all the individuals were healthy. We collected the epidemiological information by using a standardized questionnaire and collected clinical information from medical records and pathological reports.

### SNP sites selection

A total of 13 single nucleotide polymorphisms (SNPs), including eight SNPs on the gene *MMP-3* and five on the gene *MMP-8*, were selected for our study. Most of the 13 SNPs had not been reported in the past. However, several SNPs were related to some other disease, such as frozen shoulder [36], breast cancer [34], carpal tunnel syndrome [37], rheumatoid arthritis (RA) [38], or osteoarthritis (OA) [39]. The selection of SNPs depended on their location, allele frequencies, and disease relevance determined by use of the Hapmap public databases (dbSNP; http://www.ncbi.nlm.nih.gov/SNP/, HAPMAP; http://www.Hapmap.org/index.html.en). The minor allele frequency (MAF) is higher than 5% in the HapMap Chinese Han Beijing (CHB) population.

### Genotyping

We extracted genomic DNA from whole blood samples by using a purification kit (GoldMag, China), and then stored the extract at a temperature of −20° C. We measured the DNA concentration by spectrometry (DU530 UV/VIS spectrophotometer, Beckman Instruments, Fullerton, CA, USA). Per the manufacturer's instructions, we performed the genotyping by using the Sequenom MassARRAY® RS1000 system. The amplification and extension of primers were completed by application of Sequenom MassARRAY® Assay Design 3.0 software [40]. We also utilized Sequenom Typer 4.0 software to analyze and manage our data [40, 41].

### Statistical analysis

We utilized SPSS17.0 statistical software (SPSS, Chicago, IL) and Microsoft Excel to calculate the statistical analyses of our study. *P* ≤ 0.05 indicates statistical significance and all the *P*-values are two-sided. The SNP genotype frequencies in our case and control groups were performed by χ^2^ tests. We used the Hardy-Weinberg equilibrium (HWE) to check the genotype frequency of the individuals in the control group. To make sure the results of our study are credible and to assess the relation between SNPs and alcohol-induced ONFH risk, unconditional logistic regression analysis with adjustment for age was used to examined constructed 95% confidence intervals (95% CIs) and odds ratios (ORs) [42], and the adjustment for age was done for the dominant, recessive, codominant and log-additive models. In addition, we used Haploview 4.2 to test the linkage disequilibrium structure.

### Limitations

Our study had some limitations. First, patients were only enrolled in one hospital, which may increase the false-positive rate by avoiding the selection bias. This bias was not meaningful because the genetic frequencies and the difference in the distribution of demographic segmentation had been dissolved into nothingness. Second, because the number of alcohol-induced ONFH patients was not large, the sample size of our case-control study was not large. If we increase the sample size, some negative results might change to positive results that could make our conclusion more powerful and meaningful. The population was not stratified by the amount of alcohol consumption, and we did not confirm that this locus was significant for drinkers. Third, we did not evaluate the heterogeneity of alcohol consumption and the comorbidities, but in a previous study, evaluation of heterogeneity in drinking behaviors contributed to progress in elucidating the pathogenesis of alcohol-induced ONFH [43].

## CONCLUSION

We investigated 13 SNPs to explore the relation of polymorphisms of the genes *MMP-3* and *MMP-8* to alcohol-induced ONFH risk in Chinese males. We found that genetic polymorphisms of rs650108 (10556C>T) in *MMP-3* and rs2012390 (9909C>T) in *MMP-8* decreased alcohol-induced ONFH, and rs11225394 (5273G>A) on *MMP-8* with polymorphism significantly increased the risk of alcohol-induced ONFH. The mutation of the three SNPs might promote the degradation of bone matrix and influence the breakdown of extracellular matrix, the formation of osteoclasts and osteoblasts, or the activation of the inflammatory response to regulate the osteoblast/osteoclast ratio, bony tissue development, reproduction, and tissue remodeling, and then lead to the repair of bone tissue in the femoral head, and that associated with alcohol-induced ONFH risk.
